# Cost Control of Treatment for Cerebrovascular Patients Using a Machine Learning Model in Western China

**DOI:** 10.1155/2021/6158961

**Published:** 2021-11-22

**Authors:** Siyu Zeng, Li Luo, Yuanchen Fang, Xiaozhou He

**Affiliations:** Business School, Sichuan University, No. 24 South Section 1, Yihuan Road, Chengdu, China

## Abstract

**Background:**

Cerebrovascular disease has been the leading cause of death in China since 2017, and the control of medical expenses for these diseases is an urgent issue. Diagnosis-related groups (DRG) are increasingly being used to decrease the costs of healthcare worldwide. However, the classification variables and rules used vary from region to region. Of these variables, the question of whether the length of stay (LOS) should be used as a grouping variable is controversial.

**Aim:**

To identify the factors influencing inpatient medical expenditure in cerebrovascular disease patients. The performance of two sets of classification rules, and the effects of the extent of control of unreasonable medical treatment, were compared, to investigate whether the classification variables should include LOS.

**Methods:**

Data from 45,575 inpatients from a Healthcare Security Administration of a city in western China were used. Kruskal–Wallis *H* tests were used for single-factor analysis, and multiple linear stepwise regression was used to determine the main factors. A chi-squared automatic interaction detector (CHAID) algorithm was built as a decision tree model for grouping related data. The intensity of oversupply of service was controlled step by step from 10% to 100%, and the performance was calculated for each group.

**Results:**

The average hospitalization cost was 1,284 US dollars, and the total was 51.17 million US dollars. Of this, 43.42 million were paid by the government, and 7.75 million were paid by individuals. Factors including gender, age, type of insurance, level of hospital, LOS, surgery, therapeutic outcomes, main concomitant disease, and hypertension significantly influenced inpatient expenditure (*P* < 0.05). Incorporating LOS, the patients were divided into seven DRG groups, while without LOS, the patients were divided into eight DRG groups. More clinical variables were needed to achieve good results without LOS. Of the two rule sets, smaller coefficient of variation (CV) and a lower upper limit for patient costs were found in the group including LOS. Using this type of economic control, 3.35 million US dollars could be saved in one year.

## 1. Introduction

Cerebrovascular disease and its complications are the leading cause of disability and death worldwide. Of all the diseases of the nervous system, cerebrovascular diseases have the greatest impact on disability and produce the highest economic burden [1–3]. Since 2017, this disease has become the leading cause of death in China [4]. The number of people suffering from cardiovascular and cerebrovascular diseases in China was 330 million in 2019, and these diseases are the leading cause of death among urban and rural residents [5]. In 2017, the total cost of treating cerebrovascular diseases in China reached 83.83 billion US dollars, ranking first among all diseases and accounting for 17% of the total medical cost of treating diseases, equivalent to 0.66% of GDP [6]. One city alone spent 51.17 million US dollars a year on these diseases in this study. In the face of so much economic pressure, the government must take effective action to reduce the economic burden of cerebrovascular diseases.

Diagnosis-related groups (DRG) are one of the most advanced medical payment management methods, aiming to reduce inefficiency and contain costs [7]. Based on factors such as a patient's demographic information, diagnosis, and disease severity, DRG-based payment systems group patients with similar clinical attributes requiring similar care, providing the necessary framework to aggregate patients into case types or products, which entail the use of similar resources [8]. DRG adopt a standard pricing framework for a single disease group [9] and provide equity in payments across healthcare providers for services of the same kind. Most studies have found DRG to have positive effects on controlling medical expenses and reducing the economic burden among patients [10]. Studies into cerebrovascular diseases have found that DRG can effectively reduce unreasonable costs incurred in the treatment of cerebrovascular diseases [11, 12]. However, the rules of the grouping vary between countries and regions; for example, length of stay (LOS) is widely used as a statistical classification index in research into DRG management in Poland, Britain, and other developed countries [10]. Japan uses LOS as a secondary parameter [9]. However, Finland and Sweden do not consider LOS [13].

China Healthcare Security Diagnosis-Related Groups (CHS-DRG) are the unified grouping standard used by the national pilot city [14]. Due to the unbalanced development of China's economy, the Chinese government requires cities to develop localized grouping rules based on their actual conditions, so there are variations of DRG payment policy design and grouping rules across China [15]. Beijing Diagnosis-Related Groups (BJ-DRG) are the earliest localization group in China; Beijing built Chinese Diagnosis-Related Groups (CN-DRG) following the model of the All-Patient Diagnosis-Related Groups (AP-DRG) in the USA, and Shanghai built a Shanghai-DRG and National standards for paying fees according to DRG (C-DRG) based on the Australia Refined DRG (AR-DRG). However, these grouping methods are all based on the data collected from the first-tier developed cities in China, and there is no research into the underdeveloped cities in the west of the country. It is inappropriate for cities in the west to use the same rules, due to the unbalanced economic and technological development in China [16]. None of those grouping rules take into account the LOS, unlike most countries in Asia, which incorporate LOS [17].

In this study, we collected data from an underdeveloped city in western China. Machine learning was used to group patients with similar costs, and two sets of rules were built, one incorporating LOS and the other without LOS. We compared the performance of the grouping rules based on the coefficient of variation (CV) to assess the heterogeneity within a group, as has been done in previous studies [8]. We identified the outliers in each group and considered them to represent unreasonable costs. Finally, we tried to control these costs to different extents. This study fills the gap in previous studies, which have only focused on developed cities and which use CV as the standard measure of the results of grouping. In our study, underdeveloped cities and control performance were considered.

The rest of this paper is organized as follows. In Section 2, we introduce our materials and methods. In Section 3, we present our results, including general information and inpatient medical expenditure, single and multiple factor analysis of the factors influencing inpatient medical expenditure, the results of two sets of rules for DRG grouping, medical expenses in different DRG, and payment method adjustment results. In Section 4, we discuss the results.  Section 5 concludes this study and provides a description of directions for future research.

## 2. Materials and Methods

### 2.1. Patient Data

The data used in this research were collected from the Healthcare Security Administration of a city in western China during 2018. The data included medical records and cost information related to 93,185 inpatients with cerebrovascular diseases (ICD-10:60-69) as the principal diagnosis, all of which under the major diagnostic categories (MDC) of diseases and dysfunction of the nervous system (MDCB). Original information on these patients included 58 variables, such as gender, age, LOS, cost of hospitalization, payment of medical insurance, and type of insurance.

### 2.2. Data Cleaning

In the first step of data cleaning, we selected data from only the comprehensive grade tertiary and secondary hospitals. The patients from township hospitals, community hospitals, and school hospitals were removed. As a second step, we eliminated outliers in costs [8] and patients younger than 18 years of age. Finally, patients who were not hospitalized in our study city but were reimbursed by the city's Medical Insurance Bureau were excluded. Valid data from a total of 45,575 patients were obtained after screening.

### 2.3. Statistical Analysis and Data Grouping

The proportions of the training set and the test set were 80% and 20%, respectively. Firstly, the training set is grouped, and the effect of grouping is detected with the data of the test set. Finally, all the data are put into grouping rules and analyzed.

Kruskal–Wallis tests were used for single factor analysis to determine the factors influencing hospitalization expenses. Values of *P* < 0.05 were considered to be statistically significant [18]. Stepwise multiple generalized linear regression was used for variance analysis [19]. The medical costs for different subgroups were calculated, and the statistically significant variables with the greatest impacts on medical costs were selected for grouping analysis.

The Chi-Squared Automatic Interaction Detection (CHAID) algorithm was used to establish the combination of DRG [10, 20]. In the selection of grouping variables, we considered both the inclusion and exclusion of LOS, CV, and the percentage of outliers. We considered a CV value of less than 1 to indicate no heterogeneity within a group, as has been done in previous studies [8]. We regarded outliers to represent unreasonable medical treatment and calculated the variation in unreasonable medical costs among different participants under different degrees of control. We used inpatient hospitalization expenditure as the dependent variable, and the variables selected by the generalized linear stepwise model were set as the independent variables. LOS was shown to have a significant positive influence on medical expenditure. In order to further investigate the grouping performance of LOS, we built two decision tree models. The first model used the LOS as a classification variable, and the second model omitted the LOS. We have conducted more than ten random trials using data sampling samples, and the results of each trial are consistent, which indicates that the performance of the algorithm is stable. All analyses were carried out using R.studio 4.0.2 software [21] with the CHAID package [22].

## 3. Results

In the following section, we summarize general information about the patients' medical costs in Section 3.1, and single factor and multiple analysis are shown in Sections 3.2 and 3.3, respectively. The results of grouping using the two sets of rules based on machine learning are shown in Section 3.4. Finally, the performance of the algorithm using different levels of implementation control is presented in Section 3.5.

### 3.1. General Information and Inpatient Medical Expenditure

As shown in Table 1, women, individuals over 60 years old, and urban residents accounted for the majority of patients, while men, the elderly, and rural residents had relatively high expenses. Of the patients, 50.18% spent less than nine days in hospital, and 82.26% recovered after hospitalization. Of the patients with complete data, 19,488 (42.76%) were male and 26,087 (57.24%) were female; 1,995 (4.37%) were under the age of 45, while 9,117 (20%) were aged between 45 and 60, and 34,463 patients (75.64%) were older than 65. With respect to residence, 30,243 (66.36%) patients were urban workers, and 15,332 (33.64%) were rural residents. Among them, 24,482 (53.74%) were from a secondary grade hospital, and 21,087 (46.26%) were from a tertiary grade hospital. We also carried out statistical analysis on the effect of LOS, with surgery or without surgery, discharge status, and comorbidities complications (CCs) and whether there was grade III hypertension, on the distribution of patients' medical expenditure in different subgroups. The average expenditure of these patients was 1,284 US dollars. Among the subgroups, males, individuals aged over 65, rural residents, patients from tertiary grade hospitals, LOS more than 13 d, surgery, death, and CCs with insufficiency of blood supply to the cerebral arteries were more expensive.

### 3.2. Single Factor Analysis of the Factors Influencing Inpatient Medical Expenditure

In this study, 58 variables were examined using single-factor analysis (Table 1). Ten factors—gender, age, type of insurance, surgery, LOS, status on discharge, CCs, and a hypertension level of three—were shown to be associated with statistically significant differences in hospital expenditure, using Kruskal–Wallis tests (*P* < 0.01). Expenditure on men, individuals older than 60, rural residents, patients with longer LOS, patients undergoing surgery, death, and patients with CCs was the highest.

### 3.3. Multiple Factor Analysis of the Factors Influencing Inpatient Medical Expenditure

Generalized linear stepwise models were used for multiple regression analysis. Gender, LOS, level of hospital, surgery, status on discharge, type of insurance, comorbidities complications, and age had significant impacts on medical expenditure (Table 2). The *R*-squared value of the model was 0.521, and the kappa value was 12.08, indicating that the model performed well, and there was no multicollinearity between variables. All of these variables could be regarded as reasonable data for DRG grouping.

### 3.4. Two Rules for DRG Grouping and Medical Expenses in Different DRG

There were seven subgroups in model one and eight groups in model two. The hospital level was the main factor, and the second rule, without LOS, required more disease-related information, such as details of CCs. The group without LOS was more stringent. For example, grade A tertiary and grade B tertiary were in the same group under the rule incorporating LOS, while they were in different groups without LOS. The number of individuals in each group and details of expenses are shown in Tables 3 and 4. Most of the CVs of the first grouping method were less than 0.5, indicating that the homogeneity within the group was good, and the grouping effect was better in the grouping rules incorporating LOS. The weight calculation formula was (the average cost of the group)/(all the average costs). The higher the weight, the more resources consumed by the patients in the group. We set P75 + 1.5 IQR as the cost limit of each group, and the excess amount indicates the number of each group's medical expenses that were outside the cost limit.

We also analyzed the outliers of each group. Using the first grouping rules, the outliers were older than the normal patients, while using the second grouping rules, the outliers had a significantly longer LOS than the average.

### 3.5. Prediction of Medical Expenses Based on an Increasing Control Ratio of Unreasonable Treatment

In 2018, a total of 51.17 million US dollars medical expenses were related to 45,575 inpatients with cerebrovascular diseases as the principal diagnosis. The average cost was 1,248 US dollars. Among them, 43.42 million were paid by the Healthcare Security Administration, and 7.75 million were paid by patients themselves. All of this expenditure was based on the Fee for Service (FFS) payment system. We took the mean cost of each group as the payment standard for the DRG group and calculated the average cost to the Healthcare Security Administration, hospital, and patient.

The current FFS method encourages an oversupply of service in order to increase revenue [9]. We consider expenditure less than the cost limit in each group to be a normal supply and the instances in which the outliers exceed the upper limit as an oversupply of services. We increased the control intensity step by step from 10% to 100% for this oversupply service, to simulate performance under the payment system of DRG. The control effect of the two grouping rules is shown in Table 5. If we took full control, the rules with LOS could save 598,570 US dollars, and 3.35 million US dollars could be saved based on the grouping rules without LOS.

## 4. Discussion

Cerebrovascular disease has been the leading cause of death in China since 2017. The total cost of treating cerebrovascular diseases in China reached 540.6 billion yuan, ranking first among all kinds of diseases and accounting for 17% of the total cost of treating diseases, equivalent to 0.66% of GDP. Our study showed that the total cost of cerebrovascular disease was 51.17 million US dollars in an underdeveloped city in western China during 2018. The average medical expenditure on cerebrovascular disease patients was 1,284 US dollars, of which the government paid 43.42 million US dollars and patients paid 7.75 million US dollars, accounting for 84.8% and 15.2%, respectively. The government therefore paid an average of 1,087 US dollars for each patient, and each patient paid 196 US dollars for themselves. The expenditure in developed cities was even higher. Control of the medical expenses caused by cerebrovascular disease is an urgent problem for the Chinese government.

The city we chose uses a Fee for Service system, which may provide an incentive to oversupply services. We used local data to classify the patients into different groups with similar medical costs. Two models with different rules were built, based on whether the LOS was included as a classification variable. We used the CV to measure the quality of the grouping and analyzed the characteristics of the outliers in each group. We then increased the intensity of control of the oversupply of services step by step, from 10% to 100%, to simulate the performance based on the two grouping rules. The model incorporating LOS had a smaller CV than the model without LOS. If our standard model was built without LOS, it could reduce the occurrence of medical oversupply, saving 3.35 million US dollars in one year. These figures apply to only one city; if the whole country controlled costs in this way, the economic pressures on healthcare could quickly be alleviated.

Although it is generally recognized that LOS is the main factor influencing medical expenses [23], the inclusion of LOS as a classification variable of DRG is inconsistent. It is generally believed that considering LOS as a classification variable may lead to upcoding [11]. Most European countries, including England, Estonia, and Finland, do not consider LOS as a classification variable. The official Chinese CHD-DRG, modelled on the American MS-DRG, does not include LOS [14], and the Shanghai-DRG, based on the Australia AR-DRG, also does not consider LOS. However, some studies indicate that omitting LOS may increase the frequency of readmission and moves between hospitals, with services provided in alternative ways [17]. Omitting LOS also leads to poorer care for patients who should have a longer stay. The grouping rules of some countries, such as France, Ireland, and Poland, consider LOS to be an important factor [13].

Tables 3 and 4 show the results of grouping. The grouping rule with LOS has a smaller CV, indicating that the cost difference within grouping rule one was smaller, and the grouping was more reasonable. We used the P75 + 1.5 IQR as the upper limit to test for outliers in each group. The proportion of outliers was higher in the group without LOS. This observation implies that the use of LOS can lead to accurate grouping. Both grouping rules demonstrate that the hospital level is very important. In grouping rules without LOS, hospital levels and comorbidity are more finely divided. It is therefore counterproductive to consider only one hospital level.

We analyzed the outliers (Tables 3 and 4) and found that in the LOS group, the age of the outliers was significantly higher than the average value of the group, while in the group without LOS, the LOS was significantly higher than the average. A study using MS-DRG hospital data from Malta also found that most of the outliers were older and higher costs were associated with higher LOS [8]. Further analysis of these results could help identify the reasons for the high costs.

In Asia, only the Republic of Korea considers the type of hospital as a factor for DRG-based payment [9]. In this study, we found that the level of the hospital crucially influenced inpatient medical expenditure. Although there have been studies looking at the impact of hospital levels on costs [19], research into DRG has tended to focus only on tertiary hospitals. Our research therefore complements previous studies that only grouped hospitals at one level [13].

The major diagnosis was directly related to the differences in the cost of hospitalization. Comorbid patients often require special treatment and care, and different comorbidities may affect the cost of additional care, making comorbid diseases an important grouping variable. Medical costs are higher for the elderly, who require special treatments [13], but age did not show up in our grouping variables. In China, many DRG subgroups, such as the pneumonia subgroup, have age as the primary factor [19], possibly because the high cost of this group is mainly concentrated in the elderly and children. However, the age distribution of cerebrovascular disease is mainly concentrated in the elderly. In most of the European countries, like England and Estonia, age is not a factor used in grouping [13]. This observation is consistent with our findings. Most grouping rules have found surgery to be an important variable, and our single analysis also showed that surgery has a significant impact on costs. But surgery was not a variable identified in our results. This situation may have something to do with the choice of disease species. A cluster study in Beijing, China, also confirmed that in stroke, one of the cerebrovascular diseases, surgery is rare [24].

Table 5 shows the performance if the oversupply of services is controlled under the payment system of DRG. The intensity of control was increased step by step from 10% to 100%, and the results of application of the two rule sets were compared. More money could be saved without the LOS. Experience in Europe indicates that use of LOS leads to upcoding, and the medical cost was high when considering the LOS. These results imply that without LOS the cost could be controlled better, but with LOS the patients could be classified better. More incentives and oversight are needed if DRG is to be introduced. For one city, 21 million RMB could be saved by applying the results of our research, an outcome which is highly desirable for the government.

There were some limitations in this study. Due to the lack of standards for the data reported by the hospitals, there were 5,768 cases lacking information on whether surgery was performed, so these data were excluded from the grouping. Since there is no uniform surgical code between each hospital, we could not use the surgical code as our research object. Due to the large amount of data, we only considered data from one year. In the future, data from more years could be included, or the data from another year could be used for the CV of the test group.

## 5. Conclusions

We used real data from less developed regions for grouping for the DRG, filling the gap in previous studies, which took developed regions as research objects. To the best of our knowledge, this is the first time that secondary grade hospitals have been considered in a Chinese DRG study. We compared two grouping methods and discussed the results of the grouping. DRG payments were fixed, and this study adjusted the payment ratio of medical insurance, patients, and hospitals to achieve a satisfactory result for all three parties. To speed the development of DRG and rationalize the costs of cerebrovascular disease, the structure of hospital information and the standardization of data entry are essential. More research in this area is urgently needed.

## Figures and Tables

**Table 1:** Factor assignment and result of single factor analysis of the factors influencing inpatient medical expenditure (*n* = 45,575).

Variables	Assignment of influencing factors	Simple size	Expenditure $ (M + IQR)	*t*/*F*	*P* value
Gender	Male = 1	19,488 (42.76%)	1111.82 ± 741.66	247.81	<0.000
	Female = 2	26,087 (57.24%)	1026.12 ± 688.18		

Age	Age ≤ 45 = 1	1,995 (4.37%)	808.56 ± 535.69	788.16	<0.000
	Age between 45 and 60 = 2	9,117 (20.00%)	954.13 ± 640.03		
	Age ≥ 60 = 3	34,463 (75.62%)	1108.76 ± 745.46		

Level of hospital	Grade B secondary hospital = 1	7,609 (16.70%)	784.12 ± 431.26	23,064	<0.000
	Grade A secondary hospital = 2	16,879 (37.04%)	932.23 ± 671.61		
	Grade B tertiary hospital = 3	9,208 (20.20%)	1140.05 ± 825.05		
	Grade A tertiary hospital = 4	11,879 (26.06%)	1597.27 ± 1160.64		

LOS	≤9 d = 1	22,870 (50.18%)	779.17 ± 537.85	16,838	<0.000
	9∼13 d = 2	9,544 (20.94%)	1180.41 ± 884.23		
	≥13 d = 3	13,161 (28.88%)	1708.35 ± 1252.09		

Surgery	Yes = 1	2,820	1315.17 ± 765.10	330.79	<0.000
	No = 2	36,987	1013.85 ± 684.21		
	Others = 3	5,768	1212.19 ± 711.22		

Discharge status	Recovery = 1	37,492 (82.26%)	1108.33 ± 750.21	1,413	<0.000
	Transfers = 2	707 (1.55%)	933.52 ± 608.18		
	Death = 3	262 (0.57%)	1525.31 ± 760.29		
	Others = 4	7,954 (15.48%)	842.92 ± 570.62		
	Midway check-out = 5	60 (0.13%)	1112.47 ± 605.51		

Comorbidities complications	The cerebral arteries lack blood supply = 1	20,936 (45.94%)	1031.86 ± 884.13	6285.7	<0.000
	Lacunar infarction = 2	10,111 (22.19%)	1081.60 ± 740.06		
	Cerebral infarction = 3	5,246 (11.51%)	1477.85 ± 1031.87		
	Chronic cerebral ischemia = 4	1,989 (4.36%)	1089.20 ± 763.47		
	Others = 5	7,293 (16%)	1560.89 ± 974.51		

Hypertension level three	Yes = 1	9,303 (20.41)	1162.96 ± 778.03	84.216	
	No = 0	36,272 (79.59%)	1116.37 ± 699.49		

**Table 2:** Multiple linear stepwise regression results of factors influencing hospitalization expenditure in cerebrovascular disease patients.

Variables	Regression coefficient	Standard deviation	*T*-statistic	*P* value
*Gender (take the male as a reference)*				
Female	−229.84	44.53	−5.16	<0.000

*LOS (take less than nine days as a reference)*				
9 days∼13 days	2360.58	57.49	40.12	<0.000
More than 13 days	6463.63	59.93	119.86	<0.000

*Level of hospital (take grade B secondary hospital as a reference)*				
Grade A secondary hospital	1369.27	66.80	20.50	<0.000
Grade B tertiary hospital	3542.44	75.10	47.17	<0.000
Grade A tertiary hospital	6038.54	76.85	78.57	<0.000

*Surgery (take having surgery as a reference)*				
No surgery	−1480.79	90.11	−16.43	<0.000

*Status on discharge (take recovery as a reference)*				
Transfers	−669.11	265.52	−2.52	0.012
Death	3035.03	265.08	11.45	<0.000
Others	16.50	64.99	0.25	0.80
Midway check-out	−665.90	819.97	−0.81	0.416

*Type of insurance (take urban as a reference)*				
Rural	−260.14	46.82	−5.56	<0.000

*Main comorbidities complications (take cerebral arteries lack blood supply as a reference)*				
Lacunar infarction	−3814.00	67.45	−56.55	<0.000
Cerebral infarction	−3440.60	74.52	−46.17	<0.000
Chronic cerebral ischemia	−1622.16	86.57	−18.74	<0.000
Others	−3925.15	120.92	−32.46	<0.000

*Age (take less than 45 as a reference)*				
45∼60	385.83	115.15	3.35	0.001
More than 60	512.51	108.66	4.72	<0.000

**Table 3:** Results of first grouping rule (with LOS) and hospitalization expense for cerebrovascular disease patients (US dollars).

Group no.	Grouping rules	*N* (%)	Mean in US dollars	Median ± IQR	CV	Weight	Cost limit	Excess amount *N* (%)
DRG 1	Grade secondary hospital, LOS < 13 d	16,787 (42%)	760	710 ± 501	0.47	0.59	11,020	29 (1.74%)
DRG 2	Grade tertiary hospital, LOS ≤ 9 d	8,344 (21%)	1,125	1004 ± 761	0.60	0.88	15,755	282 (3.38%)
DRG 3	Grade tertiary hospital, LOS 9∼13 d	3,741 (9%)	1,620	1503 ± 1195	0.42	1.26	23,700	62 (1.66%)
DRG 4	Grade secondary hospital, LOS ≥ 13 d	5,046 (13%)	1,409	1336 ± 1043	0.36	1.09	21,044	1 (0.02%)
DRG 5	Grade tertiary hospital, CCs with the cerebral arteries lack blood supply, lacunar infarction, chronic cerebral ischemia	2,618 (7%)	2,007	1834 ± 2007	0.42	1.56	29,132	52 (1.99%)
DRG 6	Grade tertiary hospital, CCs with cerebral infarction, principal diagnosis ICD I60, I63, I65, I66, I67, I69	2,007 (5%)	2,957	2602 ± 1923	0.46	2.30	42,263	42 (2.09%)
DRG 7	Grade tertiary hospital, CCs with cerebral infarction, principal diagnosis ICD I61, I62, I64, I68	1,246 (3%)	3,368	3403 ± 2337	0.44	2.86	46,271	21 (1.68%)

**Table 4:** Results of second grouping rule (without LOS) and hospitalization expense for cerebrovascular disease patients (US dollars).

Group no.	Grouping rules	*N* (%)	Mean in US dollars	Median ± IQR	CV	Weight	Cost limit	Excess amount *N* (%)
DRG 1	Grade secondary hospital, CCs with the cerebral arteries lack blood supply, lacunar infarction, chronic cerebral ischemia	17,490 (44%)	838	773 ± 535	0.48	0.65	8,640	2,015 (11.52%)
DRG 2	Grade secondary hospital, CCs with cerebral infarction	4,343 (11%)	1,096	1001 ± 765	0.49	0.85	12,357	289 (6.65%)
DRG 3	Grade B tertiary hospital, CCs with the cerebral arteries lack blood supply, lacunar infarction, chronic cerebral ischemia	5,031 (13%)	1,203	1106 ± 735	0.51	0.94	11,852	687 (13.65%)
DRG 4	Grade A tertiary hospital, CCs with the cerebral arteries lack blood supply, lacunar infarction, chronic cerebral ischemia	5,660 (14%)	1,548	1405 ± 1063	0.47	1.21	17,142	380 (6.67%)
DRG 5	Grade B tertiary hospital, CCs with cerebral arteries supply blood, lacunar infarction, chronic ischemic cerebral, main diagnosis ICD I60, I63, I65, I66, I67, I69	2,132 (5%)	1,789	1483 ± 1048	0.63	1.39	16,980	325 (15.52%)
DRG 6	Grade A tertiary hospital, CCs with cerebral infarction, main diagnosis ICD I60, I63, I65, I66, I67, I69	2,710 (7%)	2,360	1953 ± 1187	0.67	1.84	19,147	316 (11.66%)
DRG 7	Grade B tertiary hospital, CCs with cerebral infarction, main diagnosis ICD I61, I62, I64, I68	1,172 (3%)	2,363	1983 ± 1426	0.56	1.84	22,997	430 (36.69%)
DRG 8	Grade A tertiary hospital, CCs with cerebral infarction, main diagnosis ICD I61, I62, I64, I68	1,251 (3%)	3,151	2884 ± 1746	0.57	2.45	28,160	329 (26.29%)

**Table 5:** The payment situation under different control intensity (US dollars).

			FFS	DRG control intensity									
				10%	20%	30%	40%	50%	60%	70%	80%	90%	100%
Rules with LOS	Society	Total	51.17M	51.03M	50.97M	50.91M	50.86M	50.80M	50.73M	50.67M	50.61M	50.55M	50.40M
		Average	1,284	1,282	1,281	1,279	1,278	1,276	1,275	1,273	1,272	1,270	1,263
	Hospital	Total	0	−0.06M	−0.12M	−0.18M	−0.24M	−0.30M	−0.33M	−0.42M	−0.48M	−0.54M	−0.60M
		Average	0	−1.55	−2.95	−4.50	−6.05	−7.44	−9.00	−10.54	−11.94	−13.49	−15.04

Rules without LOS	Society	Total	51.17M	50.71M	50.40M	50.09M	49.78M	49.31M	49.00M	48.69M	48.38M	48.07M	47.76M
		Average	1,284	1,275	1,267	1,258	1,250	1,242	1,233	1,225	1,216	1,208	1,199
	Hospital	Total	0	−0.33M	−0.67M	−1.01M	−1.34M	−1.68M	−2.01M	−2.35M	−2.68M	−3.01M	−3.35M
		Average	0	−8.37	−16.75	−25.27	−33.65	−42.18	−50.55	−58.93	−67.30	−75.83	−84.20

M: millions.

## Data Availability

All the data were taken from the Medical Insurance Laboratory of ChengDu Healthcare Security Administration.
